# Monitoring and Early Warning Analysis of the Epidemic Situation of *Escherichia coli* Based on Big Data Technology and Cloud Computing

**DOI:** 10.1155/2022/8739447

**Published:** 2022-02-09

**Authors:** Meishu Yan, Meizi Yan

**Affiliations:** ^1^Affiliated Hospital of Chengde Medical College, Chengde, Hebei 06700, China; ^2^Chengde Medical College, Chengde, Hebei 067000, China

## Abstract

The purpose of this study is to analyze the molecular epidemiological characteristics and resistance mechanisms of *Escherichia coli*. The study established a big data cloud computing prediction model for the epidemic mechanism of the pathogen. The study establishes the early warning, control parameters, and mathematical model of *Escherichia coli* infectious disease and monitors the molecular sequence of the pathogen based on discrete indicators. A nonlinear mathematical model equation was used to establish the epidemic trend model of *Escherichia coli*. The study shows that the use of the model can control the relative error at about 5%. The experiment proves the effectiveness of the combined model.

## 1. Introduction 

Gene promoter is the most important regulatory element of gene transcription; it determines where the gene expression starts. Therefore, the study of promoters has always been a hot spot in modern molecular biology. The theoretical prediction of gene promoters has become an important research content of bioinformatics as an important part of the identification of the complete structure of genes [1]. With the advent of the postgenomic era, although a large amount of genomic data have been generated, the available annotation information related to the promoter is still relatively scarce. Therefore, it is urgent to design a fast and effective method to identify the promoter sequence in the genome.

Because prokaryotes and eukaryotes genome promoters are quite different, they are usually studied separately for prediction. *Escherichia coli* is one of the most important prokaryotic model organisms. At present, a variety of mathematical models have been used to predict the promoter of *Escherichia coli*. The position weight matrix (PWM) is a more commonly used prediction method. Some scholars selected 288 different PWMs to conduct a systematic study on 599 sigma70 promoters. The study found that the sensitivity reached 86%, while the accuracy rate was only 53%. Some scholars have predicted 469 *Escherichia coli* promoter sequences and their positions based on predicted transcription units and using the Markov model (MM). The accuracy rate is more than 70%. The neural network method (NN) has also been used many times to predict the promoter of *Escherichia coli*. Recently, some scholars have used NNPP2.2 software to combine the distance from TSS to the translation initiation site (TIS) to improve the prediction accuracy of the *Escherichia coli* promoter [2]. Some scholars used the support vector machine (SVM) to predict 669 *Escherichia coli* sigma70 promoters and obtained high prediction accuracy. Some scholars have proposed a prokaryotic promoter identification method based on feature screening, and this method has also achieved satisfactory prediction results. We once proposed a position association scoring matrix (PCSM) algorithm to improve the prediction accuracy of promoters. Recently, some scholars have obtained higher recognition accuracy by combining the diversity increment with the secondary discriminant analysis (IDQD) method.

Although the prediction success rate of promoters is constantly improving, there are still many problems. First of all, the promoter datasets used in the past are mostly small, and the nonpromoter datasets are relatively large. This will increase the number of false positives and affect the accuracy of performance evaluation. Second, most of the work does not have a deep understanding of promoters and insufficient utilization of characteristic information [3]. Again, most of the work has carried out two predictions such as promoter and gene and promoter and coding region, and the actual need is to identify the promoter sequence from the entire genome. Therefore, such predictions lack practical significance.

In view of the problems in the prediction of the above promoters, this article will reintegrate and predict the characteristics of the promoter sequence of *Escherichia coli*. First, consider the interaction between RNA polymerase and promoter sequence. We use the position association scoring function (PCSF) to describe the positional conservation of promoter sequences. Second, the promoter sequence is divided into different windows according to the sequence characteristics, and the discrete increment index (ID) is used to measure the information content of the sequence in each window. Finally, we used the modified Markov discriminant to predict the promoter of *Escherichia coli*. Here, we call this method the IPMD algorithm [4]. Comparison with previous results shows that the algorithm we developed has better predictive performance and is more practical.

## 2. Materials and Algorithms

### 2.1. The Establishment of the Database

The *Escherichia coli* sigma70 promoter sequence is from Regulon DB, an annotation database of the *Escherichia coli* transcription regulation network. A total of 741 experimentally confirmed sigma70 promoters were obtained, and the length of each promoter sequence was 81 bp (−60…+20, TSS reference is 0 position). The negative dataset was obtained from the whole genome of *Escherichia coli* (downloaded from GenBank, sequence AC number U00096) without the promoter. But in fact, there is no experiment to prove which part of the sequence does not contain a promoter [5]. Therefore, according to the known transcription unit structure of *Escherichia coli* and the known promoter or coding region location, try to avoid regions where promoters may appear to extract negative data. The nonpromoter sequence selected in this study comes from two regions: coding region sequence and noncoding region sequence. Since the promoter drives its downstream genes, it is generally located at the head of the coding region. However, because the *Escherichia coli* genome is small, 89% are coding regions, so some promoters will exist at the end of the previous gene. Therefore, the nonpromoter of the coding region is selected in the middle part of the longer gene. Next, we select nonpromoter sequences from noncoding regions.

Based on the above considerations, we selected 700 nonpromoter and 700 nonpromoter sequences in the coding region and 700 nonpromoter sequences in the convergent region, each of which was 81 bp in length.

### 2.2. Location-Related Scoring Function

Define the standard sample set as ∑ and the position correlation weight matrix as *P*=[*p*_*xi*_]_*M*×*L*_, where *M* is the number of types of characters, *L* is the length of the sequence, and *p*_*xi*_ represents the probability of character *x* appearing at position *i*. *p*_*xi*_=*n*_*xi*_/*N*_*i*_, *N*_*i*_ is the number of the sequence, *N*_*i*_=∑_*x*_*n*_*xi*_.

Count the number of sixet fragments at each position in the sequence. We introduce the pseudocount *B*_*i*_ and redefine the matrix elements of the position association weight matrix as

(1) $$\begin{array}{c} p_{xi}=\frac{\left(n_{xi}+p_{0}\sqrt{B_{i}}\right)}{\left(N_{i}+B_{i}\right)}, \end{array}$$

where *p*_0_ is the background frequency, defined as *P*_0_=1/*N*_*i*_. We use the position weight matrix, and the associated scoring function is defined as

(2) $$\begin{array}{c} F=\sum_{i}\ln\left(\frac{P_{xi}}{P_{0}}\right). \end{array}$$

The value of *F* is used to characterize the degree of similarity between a sequence and a promoter sequence [6]. The larger the value of *F*, the more likely this sequence is a promoter sequence.

### 2.3. Discrete Increment

If there are two datasets *X* : [*n*_1_, *n*_2_,…, *n*_*s*_], *Y* : [*m*_1_, *m*_2_,…, *m*_*s*_], the discrete increment is defined as

(3) $$\begin{array}{c} \Delta \left(X,Y\right)=D\left(X+Y\right)-D\left(X\right)-D\left(Y\right)=D\left(N,M\right)-\sum_{i=1}^{s}D\left(n_{i},m_{i}\right),\\ N=\sum_{i=1}^{s}n_{i},\\ M=\sum_{i=1}^{s}m_{i},\\ D\left(N,M\right)=\left(N+M\right)\log_{b}\left(N+M\right)-N\log_{b}N-M\log_{b}M,\\ D\left(n_{i},m_{i}\right)=\left(n_{i}+m_{i}\right)\log_{b}\left(n_{i}+m_{i}\right)-n_{i}\log_{b}n-m_{i}\log_{b}m_{i}. \end{array}$$

If *n*_*i*_ or *m*_*i*_ is zero, then *D*(*n*_*i*_, *m*_*i*_)=0. It is easy to prove that the discrete increment is nonnegative, namely, Δ(*X*, *Y*) ≥ 0. We take the natural logarithm (in this case, the unit of information is knight). The discrete increment Δ(*X*, *Y*) can be regarded as a quantitative expression of the biological similarity relationship, which reflects the similarity of the two sets of data [7]. The smaller the Δ(*X*, *Y*), the more similar the two sets of data.

### 2.4. Modified Markov Discriminant

Considering samples with multiscale features, this study uses modified Markov discriminant to integrate features [8]. For any promoter sequence *S* to be predicted, the discriminant function between it and the training set can be defined as

(4) $$\begin{array}{c} \text{MD}\left(s,\mu \right)={\left(s-\mu \right)}^{T}C^{-1}\left(s-\mu \right)+\mathrm{lg}\left|C\right|. \end{array}$$

Then, the type of sequence *S* can be given by the following discriminant rules:

(5) $$\begin{array}{c} \xi =\text{MD}\left(s,\mu_{\text{pranoter}}\right)-\text{Min}\left\{\text{MD}\left(s,\mu_{\text{coding}}\right),\text{MD}\left(s,\mu_{\text{nin}-\text{coding}}\right)\right\}. \end{array}$$

Operator Min represents the smallest value in the brackets. The type of the sequence to be tested for any given threshold *ξ*_0_ can be predicted.

### 2.5. Accuracy Evaluation

We use the definitions of sensitivity (*S*_*n*_), specificity (*S*_*p*_), and correlation coefficient (CC) to evaluate the predictive performance of the algorithm.

(6) $$\begin{array}{c} \text{Senstivity}:S_{n}=\frac{\text{TP}}{\text{AP}},\\ \text{Specificity}:S_{p}=\frac{\text{TP}}{\text{AP}},\\ \text{False positive rate}:\text{FPR}=\frac{\text{FP}}{\text{AN}},\\ \text{Total accuracy}:Ac=\frac{\left(\text{TP}+\text{TN}\right)}{\left(\text{TP}+\text{TN}+\text{FP}+\text{FN}\right)}. \end{array}$$

The correlation coefficient CC=(TP∘TN − FP∘FN)/PP∘PN∘AP∘AN; the abovementioned index is used to evaluate the standard of algorithm pros and cons.

Among them, PP=TP+FP, PN=TN+FN, AP=TP+FN, AN=TN+FP.

## 3. Forecast Results

### 3.1. Promoter Feature Selection

According to the sequence characteristics of the promoter of *Escherichia coli* and the conservative analysis of its promoter sequence in the past, the characteristics of the promoter of *Escherichia coli* were selected as follows:

1. The conservative characteristic parameters of the promoter sequence. Select the sequence −51, −37, −36, −35, −34, −16, −15, −14, −13, −12, −11, −10, −9, −8, −7, −10, −2, −1 hexaplex of these 18 sites as the parameters of the positional association scoring function.
2. The component characteristic parameters of the upstream promoter sequence. We select the frequency of hexaplexes between −60 bp and −25 bp in the sequence.
3. Characteristic parameters of components near the transcription start site. We select the frequency of the hexat in the sequence between −25 bp and +21 bp.

Usually, the two-category problem has better prediction results than the three-category problem. However, because the negative data in the noncoding region and the negative data in the coding region are quite different in structure and composition, the two datasets are mixed into a negative dataset for promoter prediction research. This is bound to reduce the predictive performance of the model [9]. Therefore, the prediction model of this work will be generated by training on three datasets. The feature vector of the input modified Markov discriminant is a 9-dimensional vector (Table 1).

### 3.2. Forecast Accuracy

The prediction accuracy is the prediction ability of the test algorithm. We divide the positive sequence and the two types of negative sequence into two parts: the test set and the training set according to the ratios of 1 : 9, 2 : 8, 3 : 7, 4 : 6, and 5 : 5. In this way, the model is trained and tested [10]. The prediction results are given in Table 2. The results show that no matter what proportion of the IPMD model is trained and tested, its prediction accuracy has not changed significantly. This shows that our model is stable.

Although good prediction accuracy is obtained for various proportions of data, this test method does not fully reflect the predictive ability of the model. So next, we use a more objective 10-fold cross-check to evaluate the IPMD algorithm [11]. The 10-fold cross-check is to divide the dataset into 10 equal parts. We take one as the test set and the remaining 9 as the training set. This is repeated 10 times to test the algorithm. Then, use the receiver operating characteristic curve (ROC) to evaluate the algorithm performance. It is constructed by plotting the true positive rate and false positive rate calculated from a number of given thresholds. This is a comprehensive indicator that reflects the continuous changes in sensitivity and specificity. We use the area under the ROC curve to evaluate the prediction effect (Figure 1).

The results showed that the area under the ROC curve reached 0.953. When the optimal threshold *ξ*_0_ is selected as −1.20, the prediction sensitivity reaches 84.9% and the specificity is 84.0%. The overall accuracy and correlation coefficient are 89.2% and 0.761, respectively.

### 3.3. Comparison of Results

The above only gives the prediction results of IPMD on the three datasets. Although the overall accuracy reaches about 90%, it is not certain that our model must be better than the prediction performance of other algorithms. Therefore, according to the previous prediction methods for promoters, we carried out prediction studies on the promoter and coding region sequence and the promoter and noncoding region sequence, respectively [12–14]. We compare this algorithm with other algorithms. The 10-fold cross-check is still used here, and the comparison results are given in Table 3. Our results have been further improved compared with previous algorithm results. This can prove that the prediction model that takes into account multiple characteristics can better identify the *Escherichia coli* sigma70 promoter [15].

## 4. Conclusion

In this study, a new prediction model of the *Escherichia coli* promoter is developed. We first considered the interaction between RNA polymerase and DNA sequence and constructed a position correlation scoring function. In fact, this scoring function can roughly measure the free energy of interaction between RNA polymerase and DNA sequence. Second, the discrete index is used to describe the sequence composition of different windows of the promoter. The discrete index is another reflection form of information entropy, so the discrete increment describes the increase of sequence information. Both have strict physics meaning, but they belong to different physics concepts, which can be regarded as orthogonal in mathematics. In this way, we got the promoter description method under multiple feature scales and then used the modified Markov discriminant to realize the promoter prediction of *Escherichia coli*. The comparison with other algorithms shows that our algorithm has better performance and stronger scalability and can be extended to the promoter prediction of other species.

## Figures and Tables

**Figure 1:** ROC curve predicted by the *Escherichia coli* sigma70 promoter.

**Table 1:** Promoter feature parameter selection.

Parameter	Source of information	PCSF or ID
PCSF promoter, PCSF coding, PCSF noncoding	Hexamer frequency in eighteen conservative sites	PCSF between test sequence and promoter, coding, noncoding set
ID1 promoter, ID1 coding, ID1 noncoding	Hexamer frequency in 60 bp: −25 bp	ID between test sequence and promoter, coding, noncoding set
ID2 promoter, ID2 coding, ID2 noncoding	Hexamer frequency in 25 bp: +20 bp	ID between test sequence and promoter, coding, noncoding set

**Table 2:** The influence of different ratios on the preresults of the IPMD model.

Ratio (test set : training set)	*S*_*n*_ (%)	*S* (%)	*A*_*c*_ (%)	CC
1 : 09	85	81	88	0.735
2 : 08	82	82	88	0.731
3 : 07	82	85	89	0.754
4 : 06	81	84	88	0.732
5 : 05	78	88	89	0.744

**Table 3:** Comparison with the prediction results of other algorithms.

Method	*S*_*n*_ (×100%)	*S*_*p*_ (×100%)	CC
IPMD	95	91	0.844
	83	90	0.728

IDQD	94	83	0.75
	89	76	0.61

PCSM	91	81	0.68
	90	77	0.65

Sequence alignment kernel + SVM	82	84	0.67
	81	81	0.63

Boxes + SVM	76	83	0.62
	74	82	0.59

Boxes + threshold	76	83	0.61
	72	83	0.58

Zone likelihood + SVM	68	86	0.59
	67	84	0.56

## Data Availability

The data used to support the findings of this study are available from the corresponding author upon request.
